The article "Electroacupuncture Improves Choroidal Blood Flow to Inhibit the Development of Lens-Induced Myopia in Guinea Pigs" was published in 2022. Journal: Evid Based Complement Alternat Med.

# Electroacupuncture Improves Choroidal Blood Flow to Inhibit the Development of Lens-Induced Myopia in Guinea Pigs

**DOI:** 10.1155/2022/3286583

**Published:** 2022-06-24

**Authors:** Ting Yu, Xiaofeng Xie, Huixia Wei, Qiuxin Wu, Xiuyan Zhang, Qingmei Tian, Jike Song, Hongsheng Bi

**Affiliations:** ^1^Shandong University of Traditional Chinese Medicine, No. 16369, Jingshi Road, Jinan 250014, China; ^2^Affiliated Eye Hospital of Shandong University of Traditional Chinese Medicine, No. 48, Yingxiongshan Road, Jinan 250002, China; ^3^Shandong Provincial Key Laboratory of Integrated Traditional Chinese and Western Medicine for Prevention and Therapy of Ocular Diseases, Key Laboratory of Integrated Traditional Chinese and WesternMedicine for Prevention and Therapy of Ocular Diseases in Universities of Shandong, Eye Institute of Shandong University of Traditional Chinese Medicine, No. 48, Yingxiongshan Road, Jinan 250002, China

## Abstract

**Introduction:**

The purpose of this paper was to study the effect of electroacupuncture (EA) on choroidal blood flow (ChBF) in a guinea pig model of lens-induced myopia (LIM).

**Methods:**

Guinea pigs were randomly divided into 4 groups: normal control (NC) group, LIM group, LIM + electroacupuncture (LIM + EA) group, and LIM + sham acupoint (LIM + sham) group. Right eyes were covered with a −6D lens to induce myopia. Meanwhile, LIM + EA group and LIM + sham group were treated with EA at acupoints Hegu (LI4) and Taiyang (EX-HN5) and sham points. Refraction, axial length (AL), choroidal thickness (ChT), vessel density of choriocapillaris (CC) and choroidal layer, and scleral collagen fiber were measured. Besides, hypoxia-inducible factor-1*α* (HIF-1*α*), matrix metalloprotein-2 (MMP-2), and tissue inhibitor metalloprotease-2 (TIMP-2) expression in sclera were detected.

**Results:**

Refraction and AL were significantly decreased and ChT and vessel density of CC were significantly increased in LIM + EA group at 2 weeks and 4 weeks (all *P* < 0.05) compared with LIM group. However, no significant difference of vessel density of choroidal layer was observed between LIM and LIM + EA group at 2 weeks and 4 weeks. Scleral collagen fibrils diameters were significantly increased in LIM + EA group at 4 weeks (*P* < 0.001) compared with LIM group. At the end of experiment, the mRNA and protein expression of HIF-1*α* and MMP-2 were significantly decreased (all *P* < 0.05) and those of TIMP-2 were increased in LIM + EA, compared with LIM. However, there were no significant differences between LIM and LIM + sham group.

**Conclusions:**

EA can improve the vessel density of choroid and then possibly improve scleral hypoxia, which may inhibit the growth of the AL in myopia guinea pig.

## 1. Introduction

Myopia, which is the most common refractive disorder in the world [1], is due to the blurring of the image caused by focal plane of a distant object falling in front of the retina, resulting in the elongation of axial length [2]. At present, the prevalence of myopia is increasing. In the United States, the prevalence has increased from 25% to 44% in the last 30 years [3, 4]. In Asia, the prevalence is more than 80% [3, 5]. Therefore, it is urgent for us to define the underlying pathogenesis and to develop effective and safe therapeutic interventions for myopia.

Commonly, in mammalian eye of myopia, such as guinea pigs and mice [6, 7], it has been found that myopia is often accompanied by thinning of sclera. This is also observed in the development of myopia in humans [8]. The sclera can keep the shape and integrity of eye, and the scleral extracellular matrix (ECM) remodeling plays an important role in changing the size and refractive state of eye [9]. In 2018, Wu et al. [10] found that scleral hypoxia plays an important role in scleral ECM remodeling and participates in the development of myopia. Recently, Zhao et al. [11] have suggested that the choroid is a highly vascularized layer located between the retina and the sclera and the decrease in choroidal blood flow (ChBF) may lead to the scleral hypoxia. However, the causal mechanisms between choroid and scleral hypoxia remained largely unknown in myopia development. We suggest that myopia causes choroidal thinning and can lead to a relatively scleral hypoxic environment, and it is conceivable that such effects can result in axial elongation and myopia progression.

At present, the interventions to combat myopia progression include low-dose atropine [12, 13], MiSight contact lenses [14–16], orthokeratology lenses [17, 18], and spectacle lenses [19, 20]. In addition, EA is used to control myopia [21–23].

During electroacupuncture (EA), acupuncture needles inserted at acupuncture points and then stimulated by a device that generates electric pulses; a reformative form of the manual acupuncture is a therapeutic method in traditional Chinese medicine [24]. Acupuncture is increasingly used in the clinical treatment of many eye diseases, including dry eye syndrome [25], blepharoptosis [26], oculomotor paralysis [27], and other ophthalmic diseases [28, 29], and has a good effect. EA is also an effective method to prevent and treat diseases including angina [30], stroke [31], palpitations, [32] and coronary heart disease [33]. It is also beneficial for treating myocardial ischemia [34] and is widely used as a therapeutic technique in clinical prevention of ischemic diseases [35, 36]. Meanwhile, EA stimulation can clear blockages and increase blood flow [37–39]. This growing evidence has shown that EA pretreatment represents an important protective mechanism for tolerance against ischemia.

Therefore, we suggest that EA may increase ChBF to improve scleral hypoxia and play a vital role in the onset and development of myopia.

In the present study, we investigated the changes of ChT and ChBF in lens-induced myopia (LIM) and the expression of HIF-1*α* in sclera. Meanwhile, we observed the treatment of EA in LIM to clarify whether EA delay myopia progression by increasing ChT and ChBF to improve scleral hypoxia.

## 2. Materials and Methods

### 2.1. Animals and Experimental Design

Two-week-old pigmented guinea pigs (*Cavia porcellus*, male, 110–120 g) were supplied by the Henan Kangda Laboratory Animal Co., Ltd. They were reared under a 12-hour light/dark cycle (8 AM–8 PM) in a transparent plastic cage (20 ∗ 30 ∗ 35 cm) at 25°C with free access to fresh water and food, and the average sunlight intensity was approximately 350 lux. All experimental protocols and animal care were approved by the Animal Care and Use Committee of the Shandong University of Traditional Chinese Medicine and performed in accordance with the statement of the Association for Research in Vision and Ophthalmology (ARVO) for the Use of Animals in Ophthalmological and Vision Research [40].

80 male guinea pigs were randomly assigned to the following 4 groups (*n* = 20 per group): normal control (NC) group, lens-induced myopia (LIM) group, LIM + electroacupuncture (LIM + EA) group, and LIM + sham acupoint (LIM + sham) group. Animals in LIM, LIM + EA, and LIM + sham groups were raised with a −6D lens attached to the right eyes (Figure 1(a)). The left eyes were untreated. The lens was mounted on a home-made frame, glued onto the guinea pig's right eye with surgical tape, and cleaned every morning and evening to prevent form-deprivation myopia (FDM). Meanwhile, animals were treated with EA stimulation at acupoints Hegu (LI4) and Taiyang (EX-HN5) in LIM + EA group (Figure 1(b)) and sham acupuncture in LIM + sham group (Figure 1(c)) at the same time for 4 consecutive weeks. In our study, during the experiment, the guinea pigs underwent EA treatment under awake condition, and they have no pain or discomfort.

Electroacupuncture treatment at LI4 and EX-HN5 points and sham acupuncture was performed as previously described by Sha et al. [37]. Acupuncture needles (40 mm in length, 0.30 mm in diameter) were bilaterally inserted to a depth of 3 mm at LI4 and 2-3 mm at EX-HN5 for 30 min once a day (9:00 AM). Acupuncture needles were stimulated with an electrical stimulator (Suzhou Medical Appliance Factory of China, Model SDZ-V). The parameters were set as continuous wave electrical pulses (0.1 ms duration), frequency of 2 Hz, and intensity of 2 mA. Because low frequency is close to the frequency of manual acupuncture, 2 Hz EA stimulation is usually applied in experimental animal models for eye diseases [41, 42]. This dosage has also been verified in our group's previous myopia experiments [37], and it is the most suitable measure for guinea pigs in the awake state. Therefore, we perform EA with low-frequency EA at 2 Hz and intensity of 2 mA at the selected acupoints.

### 2.2. Biometric Measurement

In our study, we waited at least 0.5 hours and then measured refraction and AL in both eyes after EA stimulation.

Refraction was measured using streak retinoscopy. First, 1% cyclopentolate hydrochloride (Alcon, USA) was instilled into the conjunctival sac of guinea pigs every 5 min three times to reach a completely dilated pupil and cycloplegia [40]. The retinoscopy for all animals was performed by the same optometrist with a hand-held streak retinoscope (YZ24, 66 Vision Tech. Co., Ltd., China) in a dark room at 20 cm [37]. The mean value of the refraction was defined as the refractive errors of eyes, along the vertical and horizontal meridians of three repeated measurements [37, 43].

The AL was measured by A-scan ultrasonography (CineScan, Quantel Medical, France), including anterior chamber depth (VCD), lens thickness (LT), and vitreous chamber length (VCD) [44]. Before the measurement of the AL, oxybuprocaine hydrochloride (Santen Pharmaceutical, Japan) was dropped into the guinea pig's conjunctival sac and achieved topical anesthesia [40]. The tip of the probe touched the center of the cornea and was perpendicular to the plane of the cornea during the measurements. The frequency of the ultrasonic probe emission was 11 mHz. The conducting velocities were 1557.5 m/s in anterior chamber, 1723.3 m/s in lens, and 1540 m/s in vitreous chamber [44]. The AL was repeatedly measured 10 times to obtain the mean value and reduce the error.

### 2.3. Optical Coherence Tomography Angiography

For imaging, animals were prepared as previously described [45]. *In vivo* imaging of right eyes was performed with SD-OCT (Spectral-domain OCT, Spectralis HRA + OCT; Heidelberg Engineering, Heidelberg, Germany), and only images with quality values >30 were selected for further analysis [40].

#### 2.3.1. OCT Images

The enhanced depth imaging mode and the follow-up mode were firstly selected. Then, we selected OCT scans, which passed through the center of the optic disc, and the scans were exported as structural OCT images. The ChT was measured on B-scan OCT (Spectral; Heidelberg Engineering, Heidelberg, Germany). We followed the methods of Yu et al. [40].

#### 2.3.2. OCTA Images

We first selected OCTA scans which were centered on the optic disc with a field of view of 3 ∗ 1.5 mm^2^, and we acquired overlay of structural OCT and OCTA images (100% structural OCT + 100% OCTA images) [40]. The choriocapillaris (CC) was defined as the lower boundary from Bruch's membrane to less than 20 microns from Bruch's membrane [46]. The choroidal layer (medium and large vessel) was defined as the upper boundary and was less than 20 *μ*m from Bruch's membrane, and the lower boundary was set to less than 100 *μ*m from Bruch's membrane [46]. The images were imported and analyzed with ImageJ software (ImageJ, v. 1.47; National Institutes of Health, Bethesda, MD, USA). We followed the methods of Yu et al. [40, 46–48].

### 2.4. RT-PCR Examination

The scleral tissues (*n* = 3 per group) in ocular posterior poles were isolated and kept at −80°C prior to use. An RNA Tissue/Cell Rapid Extraction Kit (Sparkjade Science Co., Ltd., China) was used to extract total RNA from tissues according to the manufacturer's agreement. The RNA concentration and purity were measured using an ultraviolet spectrophotometer (K5600, Beijing Kaiao Technology Development Co., Ltd., China), and the absorbance ratio of optical density at 260 and 280 nm was 1.8–2.0 (Roche, USA). Then, synthesis of cDNA was performed using a SPARK script II RT Plus Kit (with gDNA Eraser) (Sparkjade Science Co., Ltd., China), followed by the Q-PCR amplification to determine the mRNA level with 2X SYBR Green qPCR Mix (with ROX) (Sparkjade Science Co., Ltd. China). These kits were used according to the instructions of the manufacturer. Primers were synthesized by Shanghai Sangon Biotechnology Company (Shanghai, China). The primer sequences were as follows: HIF-1*α* (200 bp): forward 5′-AGCACAACTACAGCATTCCAGCAG-3′ and reverse 5′-GGTGGTGATGTTGTGGCACGAG-3′; MMP-2 (126 bp): forward 5′-GGAATGCCATCCCTGATAACCT-3′ and reverse 5′-TTCCAAACTTCACGCTCTTGAGA-3′; TIMP-2 (118 bp): forward 5′-GAAGAGCCTGAACCACAGGTACC-3′ and reverse 5′-TTCTGTGACCCAGTCCATCCA-3′; GAPDH (170 bp): 5′-CTGACCTGCCGCCTGGAGAAACC-3′ and reverse 5′-ATGCCAGCCCCAGCGTCAAAAGT-3′. The PCR procedures were as follows: 2 min at 94°C, followed by 40 cycles of 10s at 94°C, 10s at 55°C, and 20 s at 72°C. RT-PCR was performed using a LightCycler® 480 II sequence detection system (Roche Applied Science, IN, USA). The expression levels of all genes were normalized to that of the house keeping gene GAPDH. The relative mRNA expression levels were calculated by the 2^−ΔΔCT^ method [44].

### 2.5. Western Blot

The scleras (5 scleral tissues pooled together) were covered with RIPA lysis buffer supplemented with 1 mM of PMSF in a weight to volume ratio of 1 : 10 (mg: *μ*l) and were ground under liquid nitrogen. Then, the tissue solutions were centrifuged at 4000 g·min^−1^ for 5 min at 4°C. In addition, protein concentrations were determined using a BCA Protein Assay Kit (Sparkjade Science Co., Ltd., China).

Equal amounts (50 mg) of total protein from guinea pig scleral samples were loaded onto a 12% sodium dodecyl sulfate-polyacrylamide gel, separated by electrophoresis, and electrotransferred onto a nitrocellulose membrane (Millipore, Billerica, MA, USA). After blocking with 5% nonfat milk at room temperature for 2 h, the membranes were incubated with the primary antibodies overnight at 4°C. The primary antibodies against HIF-1*α* (1 : 500, ab2185, Abcam), MMP-2 (1 : 200, Novus, NB200-113), TIMP-2 (1 : 1000, Novus, NBP2-53348), and *β*-actin (1 : 5000, Bioss, BS-0061R) were used. After washing five times for 10 minutes, each with tris-buffered saline containing Tween detergent (TBST, 10 mM Tris-HCl, pH 7.2–7.4, 150 mM NaCl, and 0.1% Tween-20), the membranes were incubated for 1 hour at room temperature with secondary antibodies. The membranes were washed again five times for 10 min in TBST. Finally, visualization was done with DAB (Sigma) by a FUSION-FX7 imaging system (Vilber Lourmat, Marne la Vallée, France), and quantification was analyzed by FUSION-CAPT software (Vilber Lourmat, France). Values were normalized to those of the *β*-actin loading control. All western blots shown are representative of at least three independent experiments.

### 2.6. Transmission Electron Microscopy Examination and Analysis

Guinea pigs (*n* = 4) from each group at 4 weeks were euthanized by injection of a lethal dose of phenobarbital sodium (130 mg/kg). A small mark was made at the 12 o'clock position on the cornea and limbus (right eye), with an indelible ink marker pen, to allow orientation of the eye cup after enucleation. Eyes were enucleated immediately after death, and the orbital fat and conjunctiva were trimmed from the eye under surgery microscope (Topcon, Japan). These eyes were fixed in 2.5% glutaraldehyde solution at 4°C for 4 h. At the end of this period, cornea and lens were dissected away, leaving the mark in the limbal region. Furthermore, a cornea trephine of 6 mm diameter was used to punch out a posterior tissue button (containing retina, choroid, and sclera). Two 2 × 1 mm^2^ strips of sclera tissue were excised from the tissue button near the nasal region, 1 mm away from the optic nerve, with razor blades [49]. The samples were further fixed at 4°C for 24–48 h and then placed in 1% osmium. After being rinsed and dehydrated in graded acetones, the tissues were embedded in an epoxy resin mixture at 60°C for 48 h. For transmission electron microscopy (Hitachi 7650, Tokyo, Japan), the scleral tissue button was equally divided into outer, middle, and inner layers (from the episclera), and five to six electron micrographs were taken from the middle layer of the sclera for each eye at x25000 [49].

The analysis of fibril diameter and density was performed by a technician. Diameters of the collagenous fibers were evaluated using an image processing software (ImageJ, v. 1.47; National Institutes of Health, Bethesda, MD, USA). The numbers that were counted ranged approximately between 100 and 300.

### 2.7. Statistical Analysis

Statistical analysis was performed using statistical software (SPSS version 22.0, Chicago, USA). Thus, our data are presented as means ± SD. Before inducing myopia, the refraction and the AL in the 4 groups showed no difference. Statistical analysis among groups was carried out using one-way ANOVA followed by an LSD post hoc test. Values of *P* < 0.05 were considered statistically significant.

## 3. Results

### 3.1. Effect of EA on the Refraction and AL

Compared with NC group, LIM group showed increased refraction, AL, LT, and VCD at 2 weeks (LIM vs. NC, refraction: *P* < 0.001; AL: *P* < 0.001; LT: *P* < 0.05; VCD: *P* < 0.01; Table 1) and 4 weeks (LIM vs. NC, refraction: *P* < 0.001; AL: *P* < 0.001; LT: *P* < 0.01; VCD: *P* < 0.001; Table 1). However, no significant difference of ACD was observed between NC and LIM group at 2 weeks and 4 weeks (all *P* < 0.05; Table 1). Compared with LIM group, LIM + EA group showed significantly decreased refraction and AL at 2 weeks (LIM vs. LIM + EA, refraction: *P* < 0.01; AL: *P* < 0.05; Table 1) and 4 weeks (LIM vs. NC, refraction: *P* < 0.001; AL: *P* < 0.05; Table 1). However, we did not detect significant changes in ACD, LT, and VCD between LIM and LIM + EA group at 2 and 4 weeks (all *P* > 0.05; Table 1). Meanwhile, there was no obvious difference between LIM and LIM + sham groups (all *P* > 0.05; Table 1). By observing the refraction and AL, we did not detect significant changes in AL compared with the fellow eyes (Tables 1 and 2).

### 3.2. Effect of EA on the Choroid

No significant differences of ChT, vessel density of CC, and vessel density of choroidal layer were observed in the 4 groups at 0 weeks (Figure 2).

Compared with NC group, LIM group showed significantly decreased ChT at 2 weeks (NC vs. LIM: 79.11 ± 7.47 *μ*m vs. 60.92 ± 8.15 *μ*m, *P* < 0.001, Figure 2(a)) and 4 weeks (NC vs. LIM: 76.38 ± 7.84 *μ*m vs. 48.43 ± 6.85 *μ*m, *P* < 0.001, Figure 2(a)). However, compared with the LIM group, LIM + EA group showed significantly increased ChT at 2 weeks (LIM vs. LIM + EA: 60.92 ± 8.15 *μ*m vs. 74.51 ± 7.07 *μ*m, *P* < 0.001, Figure 2(a)) and 4 weeks (LIM vs. LIM + EA: 48.43 ± 6.85 *μ*m vs. 73.88 ± 7.04 *μ*m, *P* < 0.001, Figure 2(a)).

Compared with NC group, LIM group showed significantly decreased CC vessel density at 2 weeks (NC vs. LIM: 28.74 ± 4.11% vs. 23.43 ± 3.85%, *P* < 0.01, Figure 2(b)) and 4 weeks (NC vs. LIM: 27.64 ± 2.91% vs. 21.29 ± 2.17%, *P* < 0.001, Figure 2(b)). However, compared with the LIM group, LIM + EA group showed significantly increased CC vessel density at 2 weeks (LIM vs. LIM + EA: 23.43 ± 3.85% vs. 27.46 ± 1.61%, *P* < 0.05, Figure 2(b)) and 4 weeks (LIM vs. LIM + EA: 21.29 ± 2.17% vs. 25.28 ± 2.39%, *P* < 0.01, Figure 2(b)).

In addition, compared with the LIM group, LIM + sham group showed non-statistically significant differences in ChT, vessel density of CC, and vessel density of choroidal layer at 2 and 4 weeks (all *P* > 0.05).

### 3.3. Effect of EA on the Scleral Collagen Fibrils

The scleral collagen fibril diameters were observed in the 4 groups at 4 weeks (Figure 2). Ultrastructural analysis revealed that the scleral collagen fibrils in NC group were wider than those in LIM group (NC vs. LIM: 82.94 ± 26.03 nm vs. 48.9 ± 23.38 nm, *P* < 0.001, Figure 2). However, compared with the LIM group, LIM + EA group showed significantly increased scleral collagen fibrils (LIM vs. LIM + EA: 48.9 ± 23.38 nm vs. 62.83 ± 21.72 nm, *P* < 0.001, Figure 2). However, no difference was found between LIM and LIM + sham groups (*P* > 0.05, Figure 2).

### 3.4. Effect of EA on the Expressions of HIF-1*α*, MMP-2, and TIMP-2 in Sclera

Compared with NC group, LIM group showed significantly increased mRNA expression levels of HIF-1*α* and MMP-2 at 2 weeks (all *P* < 0.01, Figures 3(a) and 3(b)) and 4 weeks (all *P* < 0.001, Figures 3(a) and 3(b)). The protein expression levels of HIF-1*α* and MMP-2 were increased at 2 weeks and 4 weeks (all *P* < 0.01, Figures 3(d) and 3(e)) in LIM group. However, the mRNA expression level of TIMP-2 was significantly decreased at 2 weeks (*P* < 0.01, Figure 3(c)) and 4 weeks (*P* < 0.001, Figure 3(c)) in LIM group. The protein expression level of TIMP-2 was significantly decreased at 2 weeks (*P* < 0.05, Figure 3(f)) and 4 weeks (*P* < 0.01, Figure 3(f)) in LIM group.

Compared with the LIM group, the LIM + EA group showed significantly decreased mRNA expression levels of HIF-1*α* and MMP-2 at 2 and 4 weeks (all *P* < 0.05, Figures 3(a) and 3(b)). However, the mRNA expression level of TIMP-2 was increased at 2 and 4 weeks in LIM + EA group (LIM vs. LIM + EA, *P* > 0.05, Figure 3(c)). Similarly, the protein expression levels of HIF-1*α* and MMP-2 were decreased at 2 and 4 weeks in LIM + EA group (all *P* < 0.05, Figure 3(d), 3(e)), compared with LIM group. The protein expression level of TIMP-2 was increased at 2 and 4 weeks in LIM + EA group (*P* > 0.05, Figure 3(f)).

However, the mRNA and protein expression levels of HIF-1*α*, MMP-2, and TIMP-2 were not statistically significant in LIM + sham group at 2 and 4 weeks (all *P* > 0.05), compared with the LIM group.

## 4. Discussion

In this study, we used a LIM guinea pig model to study the effects of EA on the development of myopia and found that EA plays roles in ChBF in LIM guinea pigs. During the development of myopia, we found that EA may improve scleral hypoxia by increasing the ChBF and contribute to scleral thinning, which inhibit the development of myopia in guinea pigs.

As the main oxygen source of retina and sclera, the ChBF is abundant, and the changes in ChBF are accompanied by the change of ChT. Studies [50] clearly demonstrated that the choroid could change its refractive state by modulation of its thickness. Previous studies showed that the choroid becomes thinner in guinea pigs [45]. Choroidal thinning in humans with high myopia is also associated with reductions in both its stromal and vascular components [51]. This study also demonstrates that, in chick eyes recovering from FDM, large increases in ChBF that preceded increases in ChT and were also more transient than the latter [52]. Similarly, many clinical studies have found that decreases of ChT [53, 54] and ChBF [48, 55] are associated with high myopia. The ChT and ChBF are associated with the development of myopia, which was clearly demonstrated in our studies. The choroid is a highly vascularized structure, including CC and choroidal layer (medium and large vessel). In our study, we proved that both the ChT and the vessel density of CC were decreased significantly in LIM group compared with NC group, which is consistent with the findings in previous studies [48, 56].

Meanwhile, choroid could translate visual signals and transfer them to the sclera, where they could play a role in scleral ECM remodeling and ocular growth [57]. These scleral alterations include decrease in collagen expression, myofibroblast transdifferentiation, and MMPs up-regulation as well as ECM remodeling [43]. Matrix metalloproteinases (MMPs) can degrade collagen, gelatin, and other components of ECM [58]. The proteolytic activities of MMPs are regulated by the inhibitors of metalloproteinases (TIMPs) [58]. MMP-2 and TIMP-2 could affect scleral ECM and mediate the scleral remodeling during myopia [43]. Previous studies on humans and animals have shown that MMP expression, secretion, and activity are induced by hypoxic conditions [59]. Ben et al. [60] found that activation of MMP-2 during hypoxia is associated with ECM. Importantly, HIF-1*α* in the sclera has a prominent role in signaling this restructuring, suggesting that a scleral hypoxia-dependent mechanism plays an important role in the underlying myopic development [61]. Our results showed that scleral HIF-1*α* and MMP-2 level were increased with the decrease in the ChT and the vessel density of CC in LIM group, and the scleral TIMP-2 level was decreased. At the same time, we also observed that collagen fibril diameter decreased, which is consistent with findings in previous studies [49]. Taking these findings together, we recommend that myopia-related visual signals mainly lead to a decrease in the vessel density of CC, which may lead to a decrease in the supply of oxygen and nutrients to adjacent vascular sclera.

Previous studies have reported some acupuncture related acupoints for the treatment of myopia, such as Jingming (BL1), Chengqi (ST1), Sibai (ST2), Taiyang (EX-HN5), Hegu (LI4), and Zanzhu (UB2) [23, 62–64]. In fact, clinically, EX-HN5 acupoint is often selected for the treatment of myopia [37, 65], because it is located around the eye area and EA stimulation can clear blockages and regulate the blood flow and meridians. LI4 [37, 64] is also one of the most common acupoints to be investigated in various eye diseases and the original acupoint of the large intestine meridian of Hand-Yangming, which performed desirable therapeutic effects. Sham acupuncture, also called placebo, may be considered a fake intervention, and it includes nonacupoint stimulation or insertion of acupuncture needle without rotation [66]. In our study, we performed off the sham point which was established by traditional Chinese medicine. The sham point was set at a point that was close to the lateral side of the “degenerated tail” on the gluteus muscle, a point away from the traditional meridians [67]. Therefore, we combined EX-HN5 with LI4 to observe the effect of EA on myopia in our study.

Wu et al. [10] found that two anti-hypoxia drugs, salidroside and formononetin, could delay the progression of myopia. Recently, the data strongly showed that increased ChBF can inhibit the development of myopia by attenuating scleral hypoxia [61]. It was suggested that ChBF may be a promising target for myopia retardation. In fact, EA was helpful for improving blood flow [37–39]. Previous studies have indicated that EA effectively reduced the area of myocardial ischemia and activated vascular endothelial growth factor-induced angiogenesis [68, 69]. The modulatory effect of EA on the autonomic nervous system has also been well recognized clinically [70, 71]. In fact, EA treatment could reduce infarct size by modulating sympathetic and parasympathetic nerve remodeling after myocardial ischemia, to protect the heart from further possible injury [72]. In our experiment, the ChT and the vessel density of CC in the LIM + EA group were increased more than those in the LIM group, which demonstrates the advantages of the EA in improving blood flow and improving ChBF in myopia. Furthermore, compared with the LIM group, the expressions of HIF-1*α* and MMP-2 were observed to decrease and the expression of TIMP-2 was observed to increase in sclera. These results strengthen our hypothesis that EA can improve the vessel density of ChBF and then may improve scleral hypoxia, which may inhibit the growth of the AL in myopia guinea pigs.

The choroid is mainly regulated by the sympathetic and parasympathetic nerves. Current studies have found that the choroids of mammals and birds are mainly distributed with three kinds of nerve fibers [73]: (1) parasympathetic fibers produced from the pterygopalatine ganglion (PPG) and ciliary ganglion; (2) sympathetic fibers produced from the upper cervical ganglia; and (3) sensory fibers from the trigeminal ganglion. It has been found that parasympathetic fibers are stimulated when the eye is used up close [74] and parasympathectomy prevented the development of form-deprivation-induced myopia [75]. This shows that the regulation of the parasympathetic nerve is essential during the development of myopia. PPG in mammals, which is received from the superior salivatory nucleus of the facial nuclear motor complex, innervates the choroidal vasculature and mediates vasodilation, using vasoactive intestinal peptides, acetylcholine, and nitric oxide [74]. Studies have also found that both the ciliary ganglion and the PPG affect the choroidal response to myopia defocus [75]. Therefore, we speculate that myopia stimulates the parasympathetic nerve to affect choroidal regulation and EA may improve ChBF by stimulating the parasympathetic nerve.

However, although a previous study [37] found that the level of retinal GABA, GABA_A_, and GABA_C_ receptors in LIM guinea pigs may be inhibited by EA stimulation at LI4 and EX-HN5 acupoints, it did not find that EA had obvious influence on refraction and AL of myopic eyes [37]. Experimentally, LIM had proven to be a more credible model for juvenile-onset myopia than FDM as previously reported [76], and different diopters lens were chosen in different experiments such −4D [10, 77], −6D [76], and −10D [37, 43]. We proposed that −10D lens needed more accommodation to compensate for hyperopic defocus and EA was a long and slow process that was not effective immediately. Therefore, in this study, experimental myopia was induced via −6D negative LIM to investigate the effects of EA, which can better demonstrate that EA plays a role in improving the ChBF of myopic eyes.

In addition, in our experiment, although the vessel density of choroidal layer was also improved, this was not statistically significant. It was possible that the signal attenuation of SD-OCT could not have greater depth penetration, so it was not possible to identify the detailed structure of choroid and quantify the blood flow in medium and large blood vessels. In summary, these findings indicated that EA may improve the ChBF in LIM group.

## 5. Conclusions

In summary, our results indicated that EA could improve the vessel density of ChBF and then possibly improve scleral ECM remodeling and scleral hypoxia, which may inhibit the growth of the AL in myopia guinea pigs. Moreover, these effects are observed only when EA is performed at specific acupoints. However, the effect of EA treatment on myopia still has a long way to go to explore the underlying mechanism.

## Figures and Tables

**Figure 1:** Lens-induced myopia and EA treatment experiment. (a) Lenses were mounted onto a self-made frame using surgical tapes and glued onto the right eyes of guinea pigs. (b) The guinea pigs were treated with EA stimulation. (c) The point location of acupuncture treatment (red circle).

**Figure 2:** Comparison of ChT, vessel density of CC, and vessel density of choroidal layer changes in the NC, LIM, LIM + EA, and LIM + sham group and collagen fibril diameter taken from representative electron micrographs (x25000) of the right eyes in four groups. (a) Comparison of ChT in four groups. (b) Comparison of vessel density of CC in four groups. (c) Comparison of vessel density of choroidal layer in four groups. (d) The scleral collagen fibril in NC group. (e) The scleral collagen fibril in LIM + EA group. (f) The scleral collagen fibril in LIM group. (g) The scleral collagen fibril in LIM + sham group. (d1) The corresponding distribution of the diameter of collagen fibrils in NC group. (e1) The corresponding distribution of the diameter of collagen fibrils in LIM + EA group. (f1) The corresponding distribution of the diameter of collagen fibrils in LIM group. (g1) The corresponding distribution of the diameter of collagen fibrils in LIM + sham group. ^*∗*^*P* < 0.05, ^*∗∗*^*P* < 0.01, ^*∗∗∗*^*P* < 0.001.

**Figure 3:** Changes in the HIF-1*α*, MMP-2, and TIMP-2 mRNA and protein expression during myopia development. (a) The mRNA level of HIF-1*α*. (b) The mRNA level of MMP-2. (c) The mRNA level of TIMP-2. (d) The protein levels of HIF-1*α*. (e) The protein level of MMP-2. (f) The protein level of TIMP-2. ^*∗*^*P* < 0.05, ^*∗∗*^*P* < 0.01, ^*∗∗∗*^*P* < 0.001.

**Table 1:** The refraction, AL, ACD, LT, and VCD in right eyes in groups.

Weeks	Groups	Right eyes				
		Refraction (D)	ACD (mm)	LT (mm)	VCD (mm)	AL (mm)
0 weeks	NC	3.05 ± 0.42	1.18 ± 0.03	3.34 ± 0.03	3.45 ± 0.03	7.97 ± 0.03
	LIM	3.03 ± 0.51	1.18 ± 0.03	3.35 ± 0.04	3.44 ± 0.03	7.96 ± 0.03
	LIM + LA	3.03 ± 0.49	1.19 ± 0.02	3.33 ± 0.03	3.45 ± 0.03	7.98 ± 0.04
	LIM + sham	3.05 ± 0.51	1.18 ± 0.02	3.34 ± 0.03	3.45 ± 0.02	7.97 ± 0.03

2 weeks	NC	2.2 ± 0.48	1.26 ± 0.03	3.48 ± 0.07	3.48 ± 0.06	8.22 ± 0.03
	LIM	−4.23 ± 0.43^*∗∗∗*^	1.25 ± 0.03	3.55 ± 0.05^*∗*^	3.56 ± 0.04^∗∗^	8.36 ± 0.05^*∗∗∗*^
	LIM + LA	−3.63 ± 0.49^##^	1.23 ± 0.05	3.54 ± 0.07	3.54 ± 0.04	8.32 ± 0.03^#^
	LIM + sham	−4.30 ± 0.51	1.24 ± 0.03	3.55 ± 0.04	3.57 ± 0.05	8.36 ± 0.04

4 weeks	NC	1.63 ± 0.41	1.25 ± 0.01	3.57 ± 0.05	3.58 ± 0.03	8.40 ± 0.04
	LIM	−5.88 ± 0.49^*∗∗∗*^	1.26 ± 0.05	3.65 ± 0.06^∗∗^	3.66 ± 0.04^*∗∗∗*^	8.57 ± 0.06^*∗∗∗*^
	LIM + LA	−2.55 ± 0.48^###^	1.24 ± 0.03	3.63 ± 0.05	3.64 ± 0.05	8.51 ± 0.03^#^
	LIM + sham	−5.78 ± 0.49	1.25 ± 0.02	3.65 ± 0.07	3.66 ± 0.05	8.57 ± 0.07

^+^ *P* < 0.001, LIM vs. LIM fellow; ^*∗*^*P* < 0.05, NC vs. LIM; ^∗∗^*P* < 0.01, NC vs. LIM; ^*∗∗∗*^*P* < 0.001, NC vs. LIM; ^#^*P* < 0.05, LIM vs. LIM + EA; ^###^*P* < 0.001, LIM vs. LIM + EA.

**Table 2:** The refraction, AL, ACD, LT, and VCD in left eyes in groups.

Weeks	Groups	Left eyes				
		Refraction (D)	ACD (mm)	LT (mm)	VCD (mm)	AL (mm)
0 weeks	NC	3.05 ± 0.48	1.19 ± 0.04	3.33 ± 0.02	3.45 ± 0.04	7.97 ± 0.05
	LIM	3.05 ± 0.54	1.19 ± 0.04	3.34 ± 0.06	3.42 ± 0.05	7.96 ± 0.05
	LIM + LA	3.03 ± 0.58	1.19 ± 0.04	3.35 ± 0.04	3.43 ± 0.05	7.97 ± 0.04
	LIM + sham	3.10 ± 0.49	1.19 ± 0.03	3.36 ± 0.05	3.44 ± 0.06	7.98 ± 0.05

2 weeks	NC	2.10 ± 0.43	1.27 ± 0.03	3.49 ± 0.06	3.47 ± 0.02	8.23 ± 0.02
	LIM	2.23 ± 0.53	1.27 ± 0.04	3.51 ± 0.06	3.46 ± 0.04	8.24 ± 0.03
	LIM + LA	2.23 ± 0.56	1.26 ± 0.03	3.50 ± 0.06	3.47 ± 0.06	8.22 ± 0.02
	LIM + sham	2.28 ± 0.52	1.27 ± 0.03	3.50 ± 0.05	3.49 ± 0.07	8.23 ± 0.02

4 weeks	NC	1.75 ± 0.24	1.25 ± 0.02	3.59 ± 0.07	3.56 ± 0.04	8.40 ± 0.05
	LIM	1.63 ± 0.50	1.25 ± 0.03	3.59 ± 0.05	3.58 ± 0.04	8.41 ± 0.04
	LIM + LA	1.73 ± 0.46	1.25 ± 0.04	3.58 ± 0.06	3.57 ± 0.04	8.41 ± 0.05
	LIM + sham	1.65 ± 0.36	1.27 ± 0.04	3.60 ± 0.05	3.56 ± 0.05	8.42 ± 0.06

## Data Availability

The data used to support the findings of this study are available from the corresponding author(s) upon request.
